# Influence of Sport Type on Metatarsophalangeal and Ankle Joint Stiffness and Hopping Performance

**DOI:** 10.1155/2020/9025015

**Published:** 2020-03-14

**Authors:** Yu Liu, Wing-Kai Lam, Hok-Sum Man, Aaron Kam-Lun Leung

**Affiliations:** ^1^Sports Medicine and Health School, Chengdu Sport University, Chengdu, Sichuan 610041, China; ^2^Department of Kinesiology, Shenyang Sports Institute, Shenyang 110102, China; ^3^Li Ning Sports Science Research Center, Li Ning (China) Sports Goods Company, Beijing 101111, China; ^4^Department of Biomedical Engineering, The Hong Kong Polytechnic University, Hong Kong, China

## Abstract

While individual ankle and metatarsophalangeal joint stiffness is related to training intensity and sport performances, sport athletes may develop specific passive joint stiffness among the spectrum from endurance to powerful types of sports. The objective of this study examined whether marathon runners, basketball players, and other sports athletes would demonstrate distinct passive ankle and metatarsophalangeal joint stiffness as well as vertical stiffness. Fifteen marathon runners, nineteen basketball players, and seventeen other sports athletes performed both joint stiffness measurement and single-leg hopping tests. We used a computerized dynamometer to control foot alignment and speed for passive ankle and metatarsophalangeal joint stiffness measurements. We calculated vertical stiffness by body deceleration and body mass displacement during hopping on the force platform. One-way ANOVA was performed to identify the group differences. Bivariate correlation test was also performed among ankle, metatarsophalangeal, and vertical stiffness. The basketball group displayed 13% higher ankle passive stiffness than the other sports players group (*P* = 0.03). Metatarsophalangeal joint passive stiffness in sitting and standing positions was 23% higher in the basketball group than the runner and other sports athlete groups (*P* < 0.01). However, there was no significant group differences in metatarsophalangeal joint passive stiffness and vertical stiffness. Significant correlations among all stiffness variables were determined (*P* < 0.05). These findings indicate that ankle and metatarsophalangeal joint passive stiffness, rather than vertical leg stiffness, would be in relation to types of sports participation. Ankle and toe strengthening exercises could improve basketball players' performance and prevent injury.

## 1. Introduction

Ankle and metatarsophalangeal (MTP) joint passive stiffness is extensively assessed for various sport populations in both clinical and sport settings. The ankle and MTP joint passive stiffness is related to body balance and propulsion for locomotion [1, 2]. The ankle joint connects the medial and lateral gastrocnemius muscles via the large Achilles tendon, which provides powerful plantarflexion for propulsion. It is believed that the leg muscles and the Achilles tendon can store elastic energy during the tendon elongation period and then releases energy for push/take-off during running [3] and jumping [4]. After seven-week eccentric training of lower limb muscles, the passive stiffness of the ankle joint increased by 58% [5]. The increased passive stiffness would store greater amount of elastic energy at the ankle joint for enhancing athletic performances [6–8].

The MTP joint would allow the forefoot to generate forces by pushing against the ground during propulsion of walking and running [9]. Stefanyshyn and Nigg [10] identified the MTP joint as a key foot region for minimizing energy loss during locomotion as there is little to no energy generation at the MTP joint during the push-off phase. It is speculated that a reduction in the energy dissipation at the MTP joint would lead to better running or jumping performance [10, 11]. Previous studies have suggested that the toe flexor strength (MTP passive stiffness) is positively correlated with the efficiency of walking and running [10], impact attenuation during landing [9, 12], and horizontal jumping distance [6], as well as sprinting and standing board jump [13]. Therefore, reliable measurement of the MTP joint stiffness would reflect the strength of toe flexor muscles, which has implications to toe muscle training regimes.

To date, most of the commercially available dynamometers (e.g., Biodex and Cybex), which have been used to determine strength and stiffness of the ankle joint in controlled speed and displacement [1], have limitations to use as they are bulky, expensive, and not for small MTP joints [14]. To the best of our knowledge, only manually operated dynamometer devices were recently used to measure the strength and stiffness of toes and determine the role of toe flexor muscles related to performance [6, 15, 16]. However, these dynamometers did not control the angular speed and displacement of the toe flexion and consider the alignment of the rotating axes to the anatomical of individuals, which might have caused some variations in torque measurements and limit the use of toe stiffness measurement across individuals. To date, Man and his colleagues [17] introduced a computerized ankle and MTP joint stiffness measuring device that has application before and after training treatment because it is reliable, portable, and easy to administer [14].

Since passive stiffness can be increased with training [18] and movement characteristics [16], athletes could also develop distinct passive joint stiffness according to various movement characteristics and intensity requirements in their sport participations. Compared to self-paced sports such as running, most other sports (such as basketball, soccer, tennis, badminton, and table tennis) involve a more randomized dynamic and intermittent movement pattern as they are performed at various dynamic and randomized intensities and footwork for different durations throughout match plays [19]. A stronger foot and ankle musculoskeletal structure has to be developed for these high adaptability and quick decision-making type movements [2, 18]. Furthermore, basketball players perform a large number of powerful jumps, acceleration and deceleration, lay-up, and cutting in various movement directions [20]. The increased frequent and powerful vertical jumping movements might require strong toe and ankle strength and would thus show higher passive joint stiffness in basketball athletes than the non-basketball athletes. On the contrary, runners would require optimal toe and ankle strength for better running economy [21, 22]. Studying the ankle-foot stiffness of the marathon runners, basketball players, and other athletes would help to understand how the nature of sports participation changed the mechanical properties of the human foot for adaptation.

To date, vertical stiffness (Kvert) has been predominately applied to describe the overall mechanical behaviour/efficiency of the lower extremities [23, 24] as Kvert is associated with the changes of lower extremity positions [25] and thus running economy [7]. As Kvert is influenced by lower-limb joint positions [8], it is possible that passive stiffness of the ankle joint and the MTPJ can be correlated to Kvert. Hence, the primary objective of this study was to examine whether runners, basketball players, and other sports players would demonstrate distinct ankle joint and MTPJ passive stiffness and Kvert. The second objective was to determine the correlation between Kvert and ankle/MTPJ passive stiffness. It was hypothesized that (1) basketball players might have higher joint passive stiffness for powerful jump and cut performance than other athletes and (2) Kvert might have good correlation with ankle/MTP joint passive stiffness.

## 2. Materials and Methods

Fifty-one male university team athletes were classified as long-distant runner, basketball player, and other sports players according to their participation of sports. There were 15 runners, 19 basketball athletes, and 17 other sports athletes for this study. The other sports athletes were reported to have regularly participation in different kinds of nonbasketball court sports such as table tennis, badminton, and soccer. Independent *t*-tests revealed that there were no significant differences of age, body height, body mass, and playing experience of sports between athlete groups (*P* > 0.05, Table 1). To obtain an appropriate number of participants for each group, the participants with their feet sizes from US size 7.0 to 10.0 were included in this study. All participants were free from any lower extremity injuries for the past six months prior to the start of the study. Written consent was obtained from the participants, and the testing procedure was approved by the human subject ethics subcommittee of Hong Kong Polytechnic University.

### 2.1. Passive Joint Stiffness Evaluation

The ankle and MTP joint passive stiffness was measured with a computerized dynamometer (Invention patent ZL 201410299533.4, Figure 1). In brief, the participants seated on a height-adjustable bench such that the ankle, knee, and hip joints of both legs were flexed in 90° as the starting position for both ankle and MTP joint passive stiffness measurements in the sitting position (Figure 1(a), [14, 17]). The alignment in the transverse plane and height were adjusted so that both ankle joint and MTP joint axes aligned to the rotating axis of the dynamometer by the guidance of laser line projection. During each measurement, the cradle of the dynamometer swung for 20 cycles at an angular speed of 40°/s. For MTP joint measurement, the foot was secured on a foot platform with the toes stepping out of the curved front edge so that the toes were stepping on the toe platform to measure the torque resistance (Figure 2(b)). The toes were extended by the toe plate from the neutral position (0°, horizontal) to 40° dorsiflexion (Figure 1(c)). After the MTP joint passive stiffness measurement in the sitting position was completed, the participants stood up on the dynamometer, and the MTP passive stiffness in the standing position was measured with identical foot alignment. For ankle joint measurement, the whole foot was fixed on a footplate with Velcro strap. The whole foot was periodically flexed and extended by the cradle from 20° plantarflexion to 20° dorsiflexion (Figure 1(d)). This procedure was showed to have high within-day and between-day repeatability for ankle and MTP joint stiffness [17]. The ankle and MTP stiffness had high within-day (ankle: ICC = 0.96; MTP: ICC = 0.91) and between-day repeatability (ankle: ICC = 0.96; MTP: ICC = 0.91), respectively [14].

The torque signals were smoothened by digital Butterworth zero-lag low-pass filter in the 4th-order with a cutoff frequency of 30 Hz [14, 17]. The actual ankle and MTP joint passive torques were calculated, respectively, by subtracting the torque resistance with the background torque, which was the torque resistance when the empty pedal was swinging in identical motion (Figure 2(a)). The average peak torque of middle 10 cycles (i.e., 6th to 15th cycles) was considered as the overall torque value in each trial (Figure 2(b)). The joint stiffness was the overall torque value divided by the maximum angular displacement [14, 17].

### 2.2. Hopping Performance Evaluation

Participants performed two 20-second single leg hopping on the force platform (Advanced Mechanical Technology Inc., Watertown, MA, USA) at a sampling frequency of 1,000 Hz for the left and right feet, respectively (Figure 3). The participants were required to hop with their hand placing on the hip with a frequency of 2.2 Hz using in accordance with a metronome [26]. Three-min rest between trials was allowed to minimize fatigue. The vertical reaction force was smoothened by low-pass 4th-order digital zero-lag Butterworth filter with a cutoff frequency of 10 Hz to remove the noise signal. The acceleration of center of mass (CoM) was estimated by subtracting the ground reaction force with the body weight and then divided by the body mass [3]. The displacement of CoM was then determined by double integration of the acceleration curves [3, 17]. The physical outcome was denoted by vertical stiffness (Kvert) which was calculated as the maximum reaction force divided by the maximum displacement of CoM in each hopping cycle. Kvert in each leg was the average Kvert of middle 20 hopping cycles (i.e., 11th to 30th cycles, Figure 3(b)).

### 2.3. Data Analysis

A customised MATLAB (MathWorks, Inc., Natick, MA, USA) code was applied to process all ankle stiffness, MTP stiffness, and vertical stiffness (Kvert) variables. The left and right data of each participant were averaged for further analysis. A one-way ANOVA was performed on each variable to examine if there was any significant difference between athlete groups. Additional independent-sample *t*-tests were then performed if significant athlete group effect was determined in the ANOVA. Pearson product correlation was also performed to analyse the correlation among ankle stiffness, MTP stiffness (sitting and standing), and vertical leg stiffness. The correlation (*r*^2^) was classified as little/no (>0.0 to ≤0.25), fair (>0.25 to ≤0.50), moderate to good (>0.50 to ≤0.75), and good to excellent (>0.75 to ≤1.0). All statistical analyses were conducted using SPSS version 19.0 (SPSS Inc., Chicago, IL), and the significance level was set at 0.05.

## 3. Results

The ANOVA results revealed the significant group effects for ankle passive stiffness and MTP joint passive stiffness in both sitting and standing positions (*P* < 0.01 for all comparisons) but not for Kvert (*P*=0.39). Post hoc tests indicated that both sitting and standing MTP joint passive stiffness of the basketball group were higher than the runner (*P* < 0.05) and the other sports athlete groups (*P* < 0.01) (Figures 4(a) and 4(b)). Higher ankle passive stiffness was found in the basketball group compared with the other sports groups (*P*=0.03) (Figure 4(c)).

The correlation results revealed the significant correlations among all stiffness variables (*P* < 0.01 for all comparisons, Table 2).

## 4. Discussion

Measuring ankle and MTP joint passive stiffness is extensively useful for various sport populations in both clinical and sport settings. Based on the specific movement characteristics and intensities required in different sports, athletes may develop distinct joint passive stiffness and Kvert. The present study sought to examine if runners, basketball players, and other sports players would demonstrate different ankle and MTP passive stiffness and Kvert. The present findings indicated that the basketball athletes exhibited 13% higher ankle passive stiffness than other sports athletes and that the basketball athletes demonstrated higher MTP joint passive stiffness compared to runners (sitting 24% versus standing 23%) and other sports athletes (sitting 25% versus standing 24%). A plausible explanation would be that the basketball players would require stronger toe and ankle strength as indicated by passive joint stiffness for various powerful jumping [11] and strenuous landing for better impact attenuation [9], compared with the other two tested groups who did not require frequent jumping during their sport participations.

Another possible explanation would be related to the spectrum between powerful and endurance types of performances. Distant runners may, however, require optimal toe and ankle strength/stiffness to attain the moderate speed for a long running distance [6–8]. A previous study revealed that sprinters (powerful-trained) had stiffer tendons and aponeurosis of the triceps surae compared with the long-distant runners (endurance-trained) [2], which suggested that the mechanical properties of joint stiffness are in relation to sport intensity (powerful-trained versus endurance-trained athletes). From the training perspective, eccentric exercise would increase the effective muscle length and passive muscle stiffness (i.e., titin filament), which are associated with larger force development [22] and better running and jumping performances [22, 23]. Since basketball players require stronger toe plantar flexors to adapt body balance, quick shift, and frequent jumping, further studies should identify whether more jumping/landing movements or higher movement intensity was responsible for higher joint stiffness.

The vertical stiffness (Kvert) has been commonly used to describe sports performance of different populations as it can describe the overall mechanical behaviour/efficiency of the lower extremities [23]. However, in the present study, Kvert did not show good correlations with ankle and MTP passive stiffness measurements. This could be simply explained that Kvert is influenced by musculature properties and lower extremity positions [9]. However, Kvert was not significantly different across sport types. This is contradicted to the previous findings [8], which showed that powerful-trained athletes had higher leg stiffness than the endurance-trained athletes. The contradicting results would be explained by the compensation related to individual joint movements and muscular properties. In the future, comparing ankle and MTP joint stiffness may have better discriminative ability to identify the talent for basketball players, especially in the fatigue situation [27].

The previous ankle and MTP passive stiffness measurements are still largely depended on manual skills as the previous devices did not have good control on alignment, angular speed, and displacement during torque measurements [15]. In the present study, we measured the ankle and MTP joint passive stiffness measurements with the computerised dynamometer, which would provide good control of alignment, angular joint speed, and displacement [14, 17]. While both sitting and standing MTP stiffness findings demonstrated the similar trend across athlete groups, higher MTP stiffness values were observed in the standing posture compared with the sitting posture. During standing, plantar aponeurosis was tightened, contributing to higher MTP stiffness values. This suggests that the MTP passive stiffness would be related to the weight bearing and joint positions. In practical application, MTP stiffness measurement is recommended to be performed in the sitting position as it has similar discriminative ability (Figures 4(a) and 4(b)), better relationship level with ankle stiffness (Table 2), and easy to posture control [16, 17]. The findings of our study would facilitate the understanding of sports performances and the development of treatment and rehabilitation protocols in ankle and forefoot injuries. In footwear application, optimising forefoot bending stiffness (at the MTP region) could enhance jumping, sprinting, and agility performance [11, 28]. Additionally, joint contact force can provide additional information for better estimation of knee joint loading during movements [29]. In training application, optimising ankle and MTP joint stiffness could also improve running pattern and minimise the risk of injuries [30]. Monitoring MTP joint stiffness could be a mean to evaluate surgical and rehabilitation (intensity and duration) outcomes in forefoot-related injuries [7, 25].

There are some experimental limitations when interpreting our results. Firstly, a single male university athlete group was recruited in this study, and it is not generalizable to other groups. Different genders, playing levels, and positions may have shown remarkable differences in jumping intensity and frequency in match plays [20]. Secondly, only joint stiffness data were examined in the present study, and therefore, interpretation of the findings with sports performance has to be prudent. Future studies can consider a more comprehensive evaluation including measurements of sport performance (e.g., jump, run, and agility) and muscular activity.

## 5. Conclusions

Basketball athletes displayed higher ankle and MTP joint passive stiffness compared with distant runners and other sports athletes, suggesting that mechanical properties of joint stiffness are in relation to sport intensity between powerful- and endurance-trained athletes. Ankle and toe strength exercises could be implemented to develop sufficient ankle and MTP joint passive stiffness that is required in basketball.

## Figures and Tables

**Figure 1:** The ankle and MTP joint stiffness measurement device: (a) experimental setup and MTPJ axis alignment with a laser beam, (b) the foot and toe platform components, (c) illustration of ankle passive stiffness measurement, and (d) illustration of MTP joint passive stiffness measurement.

**Figure 2:** (a) Illustration of net joint torque measurement and (b) raw and net joint torque against time.

**Figure 3:** (a) Illustration of hopping performance and (b) raw and net vertical stiffness against time.

**Figure 4:** (a) MTP passive stiffness in standing, (b) MTP passive stiffness in sitting, (c) ankle passive stiffness, and (d) vertical stiffness.

**Table 1:** Mean (SD) and *P* values between sport types.

	Runner	Basketball athlete	Other athletes	*P* value
Age (yr)	22.7 (2.3)	21.7 (1.8)	22.9 (2.8)	0.272
Height (m)	1.74 (0.06)	1.77 (0.06)	1.74 (0.07)	0.252
Mass (kg)	67.9 (8.1)	71.2 (6.1)	67.2 (6.8)	0.202
Playing experience (yr)	5.7 (4.2)	5.7 (2.2)	3.8 (2.9)	0.123

**Table 2:** Pearson correlation (*r*^2^) and *P* values between stiffness variables. Significant *P* values (*P* < 0.05) are shown in bold.

	*P* value	*r* ^2^	Relationship level
Ankle stiffness vs. MTPJ stiffness (sit)	**<0.001**	0.51	Moderate to good
Ankle stiffness vs. MTPJ stiffness (stand)	**<0.001**	0.24	Little/no
Ankle stiffness vs. vertical stiffness	**<0.001**	0.15	Little/no
MTPJ stiffness (sit) vs. MTPJ stiffness (stand)	**<0.001**	0.53	Moderate to good
MTPJ stiffness (sit) vs. vertical stiffness	**<0.001**	0.15	Little/no
MTPJ stiffness (stand) vs. vertical stiffness	**<0.001**	0.06	Little/no

## Data Availability

The data used to support the findings of this study are available from the corresponding author upon request.
